# Quality Prediction of Fused Deposition Molding Parts Based on Improved Deep Belief Network

**DOI:** 10.1155/2021/8100371

**Published:** 2021-12-07

**Authors:** Hai Dong, Xiuxiu Gao, Mingqi Wei

**Affiliations:** ^1^School of Applied Technology, Shenyang University, Shenyang 110041, China; ^2^School of Mechanical, Shenyang University, Shenyang 110041, China

## Abstract

Tensile strength, warping degree, and surface roughness are important indicators to evaluate the quality of fused deposition modeling (FDM) parts, and their accurate and stable prediction is helpful to the development of FDM technology. Thus, a quality prediction method of FDM parts based on an optimized deep belief network was proposed. To determine the combination of process parameters that have the greatest influence on the quality of FDM parts, the correlation analysis method was used to screen the key quality factors that affect the quality of FDM parts. Then, we use 10-fold cross-validation and grid search (GS) to determine the optimal hyperparameter combination of the sparse constrained deep belief network (SDBN), propose an adaptive cuckoo search (ACS) algorithm to optimize the weights and biases of the SDBN, and complete the construction of prediction model based on the above work. The results show that compared with DBN, LSTM, RBFNN, and BPNN, the ACS-SDBN model designed in this article can map the complex nonlinear relationship between FDM part quality characteristics and process parameters more effectively, and the CV verification accuracy of the model can reach more than 95.92%. The prediction accuracy can reach more than 96.67%, and the model has higher accuracy and stability.

## 1. Introduction 

Additive manufacturing (AM) is a rapid prototyping technology born in the 1980s, which realizes the conversion from a 3D digital model to a physical model by continuously adding layers of materials. Compared with traditional subtractive manufacturing (cutting), additive manufacturing has the characteristics of energy-efficient, green, and recyclable [1–3], which meets the market demand for rapid product development and personalized customization. Fused deposition modeling (FDM) has become one of the most widely used additive manufacturing technologies at home and abroad because of its simple molding equipment, low production cost, and the ability to manufacture complex parts without extra tools [4, 5]. At present, fused deposition molding has been widely used in consumer products, automobiles, aerospace, and medical and construction fields and has achieved huge economic benefits; however, FDM technology still faces challenges. In the process of rapidly preparing parts in the fused deposition process, the material undergoes three stages of solid phase, molten state, and cooling and solidification. In this process, the mechanical properties of raw materials, changes in the forming temperature field, and process forming parameters all have an impact on the quality of the parts [6–9]. The main quality problems of FDM parts include poor tensile strength, warpage deformation, and insufficient surface accuracy. These problems hinder the development of the fused deposition process in industrial production and become a key issue that needs to be solved urgently in the development of the additive manufacturing industry.

To solve the above problems, much research focuses on understanding and optimizing FDM process parameters to enhance the performance characteristics of products and expand the application fields of FDM technology. Wang et al. [10] modeled the warpage deformation printed parts, which considered the material properties and machine settings of FDM, such as layer thickness, printing path, extrusion temperature, and speed. They pointed out that the warpage deformation could be effectively reduced by improving the temperature and printing path. Nancharaiah et al. [11] studied the effects of grating angle, layer thickness, and width on the surface roughness of FDM parts by using the Taguchi method and ANOVA technique. The experimental results have shown that layer thickness significantly affects the accuracy of FDM parts. Sahu et al. [12] et al. analyzed the influence and interaction of process variables such as layer thickness, printing direction, grating angle, grating width, and air gap on the surface accuracy of parts. Mohamed et al. [13] proposed the optimal standard for optimizing the process parameters of FDM and studied the nonlinear relationship between the process parameters and dimensional accuracy. Zaman et al. [14] and Dev et al. [15] designed experiments based on Taguchi's method and studied the influence of process parameters on the tensile strength of FDM parts. Tura et al. [16] established a mathematical prediction model of controllable input parameters using the response surface method to explore the influence of FDM input parameters on the surface roughness of ABS materials. Although traditional quality methods and mathematical modeling can verify the influence of process parameters on a certain performance of FDM parts, it is difficult to accurately establish the mapping relationship between input variables and output variables, so the improvement effect on product quality is not obvious.

The data-driven prediction method has been widely used in recent years due to its strong adaptability [17]. As a typical data-driven method, machine learning constructs an approximate model based on real-time, historical, and relational data to approach the real situation and build a prediction model. As an important branch of machine learning, the neural network has been applied to product performance prediction due to its powerful data and nonlinear processing capability [18–21]. Therefore, some literature constructed quality prediction models to realize the prediction of FDM parts quality. To improve the surface roughness of FDM parts, Vahabli and Rahmati [22] built a surface roughness distribution model and proposed a prediction method of product surface roughness based on the radial basis function neural network (RBFNN). Zhang et al. [23] proposed the FDM parts quality prediction model based on the long-short term memory network (LSTM) to predict the tensile strength of parts. Ali and Chowdary [24], Pazhamannil et al. [25], and Manoharan et al. [26] all used the artificial neural network (ANN) model to predict the tensile strength of FDM parts. Zhang and Yang [27] used the genetic algorithm to optimize the weights and thresholds of the BP neural network (BPNN) and established a precision prediction model for FDM parts based on process parameters. All the above prediction methods are shallow machine learning models. Although these methods can be used to predict the roughness, warping degree, or tensile strength of FDM parts, they cannot adequately extract the effective features of training samples, and it is difficult to accurately map the complex nonlinear relationship between multiple process parameters and multiple quality indicators, and the model has poor stability.

Deep belief network (DBN) is a deep neural network composed of several restricted Boltzmann machines (RBMs). Compared with the neural network with a single hidden layer structure, the DBN has better ability of feature learning and nonlinear fitting. At present, various deep learning models based on the DBN are widely used to solve many challenging problems, such as quality prediction [21, 28], fault diagnosis [29], flow prediction [30, 31], wind energy prediction [32], image classification [33], prediction of concrete compressive strength [34], and air quality assessment [35]. The feature information extraction of the DBN depends on the RBM. Inspired by the sparse representation of visual cortex, the sparse concept is introduced into the RBM to facilitate the upper neurons to extract the most essential features in the stimulation and learn more effective feature information. Experiments show that the sparse deep belief network (SDBN) formed by sparse limited Boltzmann mechanism (SRBM) can extract feature information more effectively and avoid the problem of model overfitting [36]. In addition, the above literature shows that the network parameter setting of the DBN has a significant impact on the model performance. There are two types of parameters in the DBN model. The first type is the value set before the model starts the learning process, such as the model learning rate, the number of hidden layers, and the number of hidden elements. These parameters are called superparameters. The second category is the parameters obtained by the model through learning and updating, such as weights and bias. This study is based on the grid search method to determine the optimal hyperparameter combination of the sparse deep belief network model. There are few studies on DBN hyperparameter optimization, and researchers mostly use empirical methods to solve the problem of the network structure [37], In this article, the grid search (GS) method is used to search all possible combinations of the SDBN model's hyperparameters, and the best combination of the model's hyperparameters is determined by taking the validation error value of 10-fold cross-validation as the evaluation standard. For weights and thresholds, heuristic algorithms are often used to optimize [38]. Moreover, the prediction performance of the neural network optimized with weights and thresholds is obviously better than that of the single neural network without optimization [39]. Based on this, this article proposes an adaptive cuckoo search (ACS) algorithm to optimize the learning parameters of the SDBN. The significant advantage of the ACS algorithm is that it involves fewer codes and parameters and has a strong global search capability.

The motivation of this research is to use a new prediction model, which takes FDM process parameters as model input, to realize the accurate prediction of the three quality characteristics of FDM parts, namely, tensile strength, warping degree, and surface roughness. The GS-ACS-SDBN prediction model proposed in this article is based on deep learning, and uses GS and 10-fold cross-validation to determine model hyperparameters and the ACS algorithm to optimize model weights and biases. Compared with the prediction results of the DBN, LSTM, RBFNN, and BPNN models, the GS-ACS-SDBN model has more sufficient learning of data features and can achieve accurate prediction of the quality of FDM parts. The experimental results are successful and proved the effectiveness of this method.

The main contributions and innovations of this study are as follows: firstly, we construct a new quality prediction model, which can predict the roughness, warpage, and tensile strength of FDM parts at the same time; secondly, the optimal learning rate, the number of hidden layers, and the number of hidden elements of the SDBN model are determined by grid search and cross-validation, and this method can realize the automatic selection of model parameters; finally, an adaptive cuckoo search algorithm is proposed by introducing the cosine diminishing strategy, and the algorithm is used as the optimizer of the model to improve the prediction accuracy of the model. In addition, we discuss the performance of the GS-ACS-SDBN prediction model.

The rest of the article is organized as follows: in Section 2, we introduce the ACS algorithm and SDBN. In Section 3, we propose an FDM part quality prediction method based on the GS-ACS-DBN model and compare the prediction results of the GS-ACS-SDBN with other prediction models to verify the superiority of our method. The conclusions are discussed in Section 4.

## 2. Sparse Deep Belief Network and Adaptive Cuckoo Search

### 2.1. Sparse Deep Belief Network Model Construction

DBN is a probability graph model composed of several RBMs. DBN training adopts the strategy of greed layer by layer, and the output of the RBM of each layer is used as the input of the next layer. Its structure is shown in Figure 1.

RBM is composed of multiple hidden layer neurons and multiple visible layer neurons. The former layer neurons are used for training data, whereas the latter layer neurons are used for feature extraction. The probability of activation of neurons in the visible layer (*v*) and the hidden layer (*h*) is 0 or 1, and they are connected in a bidirectional equal weight mode; the weight is *w*_*i*,*j*_, and the neurons in the same layer are independent of each other. *a*_*i*_ and *b*_*j*_ represent the paranoid threshold of the visible layer and the hidden layer, respectively.

The probability distribution of the RBM can be realized by the energy function, which is defined in the given state (*v*, *h*) as

(1) $$\begin{array}{c} E_{\theta }\left(v,h\right)=-\sum_{i=1}^{n}a_{i}v_{i}-\sum_{j=1}^{m}b_{j}h_{j}-\sum_{i=1}^{n}\sum_{j=1}^{m}v_{i}w_{ij}h_{j}. \end{array}$$

After visualization and regularization of the above equation, the joint probability distribution of the RBM can be obtained as shown in the following equation:

(2) $$\begin{array}{c} P\left(v,h;\theta \right)=\frac{1}{z\left(\theta \right)}\exp\left(-E_{\theta }\left(v,h\right)\right), \end{array}$$

where *z*(*θ*) is a normalized factor, expressed as

(3) $$\begin{array}{c} z\left(\theta \right)=\sum_{v,h}\exp\left(-E_{\theta }\left(v,h\right)\right), \end{array}$$

where *θ*={*w*_*ij*_, *a*_*i*_, *b*_*j*_} is the network parameter. When the visual layer vector *v* is given, the probability that the hidden layer neuron *j* will be activated is

(4) $$\begin{array}{c} P\left(h_{j}=1|v\right)=R\left(\sum_{i=1}^{n}w_{ij}v_{i}+b_{j}\right). \end{array}$$

The probability of visual layer vector neuron *i* being activated is

(5) $$\begin{array}{c} P\left(v_{i}=1|h\right)=R\left(\sum_{j=1}^{m}w_{ij}h_{j}+a_{i}\right), \end{array}$$

where *R* represents ReLU activation function, which is used to activate neurons. It has a better feature learning ability than Tanh activation function and sigmoid activation function. The updating rules of parameters are shown in the following equations:

(6) $$\begin{array}{c} w_{ij}^{t+1}=w_{ij}^{t}+\varepsilon \left({\langle v_{i}h_{i}\rangle }_{\text{data}}-{\langle v_{i}h_{i}\rangle }_{\text{rec}}\right), \end{array}$$

(7) $$\begin{array}{c} a_{i}^{t+1}=a_{i}^{t}+\varepsilon \left({\langle v_{i}\rangle }_{\text{data}}-{\langle v_{i}\rangle }_{\text{rec}}\right), \end{array}$$

(8) $$\begin{array}{c} b_{j}^{t+1}=b_{j}^{t}+\varepsilon \left({\langle h_{j}\rangle }_{\text{data}}-{\langle h_{j}\rangle }_{\text{rec}}\right), \end{array}$$

where *ε* is the learning rate; < >_data_ represents input data; and < >_rec_ represents reconstructed data.

The feature information extraction of the DBN depends on the RBM. Inspired by the sparse representation of the visual cortex, the sparse concept is introduced into the RBM to facilitate the upper neurons to extract the most essential features in the stimulation and learn more effective feature information. Lorentz function sparse constraint has been applied in many fields such as detection and image discrimination, and relevant experiments show that this method can effectively extract feature information and suppress environmental noise [40].

We use *l*_*s*_ to represent the Lorentz measure of sparsity and *S* to represent the controlling factor of activation probability sparsity. To obtain the sparse representation of the model in the learning process, weight and threshold need to be adjusted so that the RBM can maximize the likelihood function and obtain the sparse distribution of the training set. The objective function of the SRBM model is as follows:

(9) $$\begin{array}{c} \ln\;l_{S}=\min\left\{w_{ij},a_{i},b_{j}\right\}-\sum_{k=1}^{K}\log\left(\sum_{t}p\left(v_{i}^{k},h_{j}^{k}\right)\right)\\ +\lambda \sum_{k=1}^{K}\sum_{j=1}^{m}\log\left(1+\frac{{\left(E\left[h_{j}^{k}|v_{i}^{k}\right]\right)}^{2}}{S^{2}}\right). \end{array}$$

In the above equation, the second term is the likelihood term and the third term is the regularization term. *l*_*S*_ represents the Lorentz metric of sparsity, *S* represents the control factor of the sparsity of activation probability, *k* represents the *k*-th layer, *k* ∈ *K*, and *λ* is the regularization parameter. The SRBM training uses the contrast divergence algorithm to obtain the approximate gradient of the likelihood term and solve the regular term. The gradient calculation process of the regular term is shown in the following equations:

(10) $$\begin{array}{c} \frac{\partial }{\partial w_{ij}}l_{S}=\sum_{k=1}^{K}\frac{\partial }{\partial w_{ij}}\log\left(1+\frac{{\left(E\left[h_{j}^{k}|v_{i}^{k}\right]\right)}^{2}}{S^{2}}\right)=\sum_{k=1}^{K}\frac{2p^{k}}{S^{2}+{\left(p^{k}\right)}^{2}}p^{k}\left(1-p^{k}\right)v_{i}^{k}, \end{array}$$

(11) $$\begin{array}{c} \frac{\partial }{\partial b_{j}}l_{S}=\sum_{k=1}^{K}\frac{\partial }{\partial b_{j}}\log\left(1+\frac{{\left(E\left[h_{j}^{k}|v_{i}{}^{k}\right]\right)}^{2}}{S^{2}}\right)=\sum_{k=1}^{K}\frac{2p^{k}}{S^{2}+{\left(p^{k}\right)}^{2}}p^{k}\left(1-p^{k}\right). \end{array}$$

### 2.2. Data Sampling Based on Gibbs

Gibbs sampling is based on the sampling method of Monte Carlo–Markov chain, and its basic theory is similar to the Metropolis algorithm. Assuming that the dimension of the existing sample is *N*, the mathematical expression of the sample is given as *X*=(*x*_1_, *x*_2_,…, *x*_*n*_), assuming that the overall distribution of the sample *P*(*x*)) is unknown, but other variables other than *x*_*i*_ are known, the conditional distribution probability of sample xi can be obtained, that is, *P*(*x*_*i*_/*x*_*i*−_) (*x*_*i−*_ means that the variable *x*_*i*_ is removed from the sample as a whole). In addition, for any state of *x*, it is set as [*x*_1_^(0)^, *x*_2_^(0)^,…, *x*_*n*_^(0)^], and the remaining variables are sampled based on the conditional probability distribution formula, and the number of sampling increases with the number of iterations. After *t* sampling, the distribution of the sample states [*x*_1_^(*t*)^, *x*_2_^(*t*)^,…, *x*_*n*_^(*t*)^] will converge to the global distribution at the geometric speed of *t*.

The specific sampling process is as follows:

(12) $$\begin{array}{c} v_{1}∼P\left(v\right),\\ h_{1}∼P\left(h|v_{1}\right),\\ v_{2}∼P\left(v|h_{1}\right),\\ h_{2}∼P\left(h|v_{2}\right),\\ \ldots \\ v_{t+1}∼P\left(v|h_{t}\right). \end{array}$$

Given the state of visual layer neurons in the RBM, the state of hidden layer neurons can be reconstructed:

(13) $$\begin{array}{c} h=\text{sample }h\text{ given}\left(\begin{array}{c} v\;\text{RBM} \end{array}\right). \end{array}$$

Given the state of hidden layer neurons in the RBM, the state of visual layer neurons can be reconstructed:

(14) $$\begin{array}{c} v=\text{sample }v\text{ given}\left(\begin{array}{c} h\;\text{RBM} \end{array}\right). \end{array}$$

### 2.3. Model Pretraining

Unsupervised learning is used to pretrain the DBN and provide a better parameter basis for further parameter fine-tuning. In the process of mixed pretraining, to ensure the integrity of the prediction model, a temporary output layer should be stacked on the RBM to be trained.

In unsupervised training, the model needs to seek reconstructed data $\hat{m}$ close to the original data *m*, namely,

(15) $$\begin{array}{c} \left\|\hat{m}-m\right\|⟶0. \end{array}$$

We selected *M* training samples, defined *f*_*i*_ as the predicted value and *F*_*i*_ as the true value, and calculated the reconstruction error function *C*:

(16) $$\begin{array}{c} C=\text{MAE}=\frac{1}{M}\sum_{i=1}^{M}\left|f_{i}-F_{i}\right|. \end{array}$$

After layer by layer mixed pretraining, the BP algorithm is used to fine-tune global parameters. The BP neural network has good information forward transmission and error back propagation characteristics. Through repeated cycles to achieve the desired error, finally after training to get the desired model.

The training steps of the RBM are given as follows:

### 2.4. Aaptive Cuckoo Search

CS algorithm is a new intelligent optimization algorithm proposed by Yang and Deb in 2009. The significant point of this algorithm is that it adopts Levy flight mechanism to conduct search. Levy flight is a random search method that combines short-frequency long-distance flight and high-frequency short-distance flight to realize random jump search in different areas, which effectively balances the local search and global search capabilities of the algorithm [41]. Levy's flight path is shown in Figure 2.

Based on the general principle of cuckoo search, the optimization ability of cuckoo depends on two aspects: (1) the step size control factor *α*, whose value determines the contraction range of Levy's flight, and (2) discard probability *p*_*a*_, the value of *p*_*a*_ determines the number of new nests retained, namely, the diversity of the population. In the standard cuckoo search algorithm, *α* and *p*_*a*_ are fixed values, which cannot well adjust the step size generated by Levy's flight and ensure the diversity of the population. For this reason, we adopt the decreasing cosine strategy [42] to realize the dynamic and adaptive change of step size.

The expression of adaptive discarding probability is as follows:

(17) $$\begin{array}{c} p_{a}=p_{a,\max}\cos\left(\frac{\pi }{2}\cdot \frac{t-1}{t_{\max}-1}\right)+p_{a,\min}. \end{array}$$

The expression of the adaptive step size control factor is as follows:

(18) $$\begin{array}{c} \alpha^{t}=\left\{\begin{array}{c} \alpha_{\max}\cos\left(\frac{\pi }{2}\cdot \frac{t-1}{t_{\max}-1}\right),\;R\leq a,\\ \alpha^{t-1}\left(\frac{\pi }{2}\cdot \frac{t-1}{t_{\max}-1}\right),\;a<R\leq b,\\ \alpha_{\min}\left(\left(\frac{\pi }{2}\cdot \frac{t-1}{t_{\max}-1}\right)\right),\;R>b, \end{array}\right. \end{array}$$

where *R* is the iteration ratio, *R* = *t/t*_max_; and *a* and *b* are constants, *a*, *b* ∈ (0,1).

The bird's nest position update method based on the dynamic adjustment strategy is further defined as

(19) $$\begin{array}{c} x_{i}^{t+1}=\left\{\begin{array}{cc} x_{i}^{t}+\left[\alpha^{t}\cdot \left(x_{i}^{t}-x_{\text{best}}^{t}\right)\right]⊕\text{Levy}\left(\beta \right)\text{ if }, & P\geq p_{a},\\ x_{i}^{t}, & P<p_{a}. \end{array}\right. \end{array}$$

The optimization process of the ACS algorithm shown as follows:

## 3. FDM Parts Prediction Method Based on GS-ACS-DBN

The main process of FDM parts quality prediction includes key quality factor screening, GS-ACS-SDBN prediction model construction, and FDM parts quality prediction. The quality prediction process of FDM parts based on the GS-ACS-SDBN model is shown in Figure 3.

### 3.1. Key Quality Factor Screening

FDM image files are usually stored as STL files. The computer processes the image files in layers and determines the path of material deposition layer by layer. The wire feeder feeds the wire to the nozzle, where the wire is heated and melted to a molten state. The wire flows out of the nozzle and moves along a predetermined print path to deposit the molten material. The extruded material then cools and forms a single layer. Once the first layer is finished, the support platform lowers the predetermined distance to allow the deposition of the higher layers, which continues until the product is printed. The forming process of FDM parts is shown in Figure 4.

In this article, I font with length, width, and height of 150 mm, 30 mm, and 5 mm, respectively, is used as the printing pattern, as shown in Figure 5. The experimental equipment is Aurora Irva Z-603S, and the experimental consumables are ABS materials and PLA materials. Pattern printing takes the origin as the starting point for horizontal printing, and the filling density is 100%. The process parameters include slice thickness, extrusion speed, nozzle temperature, and molding room temperature. The parameter setting range is shown in Table 1; the performance parameter information of ABS and PLS materials is shown in Table 2. Based on the orthogonal printing method, 2500 valid samples were obtained, among which 80% samples were taken as the training set and the remaining 20% as the test set.

Data correlation testing helps to determine the main factors affecting product quality and to improve the prediction results. For this reason, the article uses the combinational correlation test method (RV_mod_), proposed by Smilde et al. [43], to calculate the correlation degree between each FDM process parameter and quality characteristics. RV_mod_ is the generalization of correlation analysis such as multiple regression analysis, principal component analysis, and canonical correlation analysis. The calculation formula is as follows:

(20) $$\begin{array}{c} \left\{\begin{array}{c} {\text{RV}}_{\mathrm{mod}}=\frac{\text{tr}\left(AB\right)}{\sqrt{\text{tr}{\left(A\right)}^{2}\text{tr}{\left(B\right)}^{2}}},\\ A=XX^{T}-\text{diag}\left(XX^{T}\right),\\ B=YY^{T}-\text{diag}\left(YY^{T}\right), \end{array}\right. \end{array}$$

where *X* represents the matrix of influencing factors, including the process parameters in Tables 1 and 2; and *Y* is the product quality characteristics, including surface roughness, warping degree, and tensile strength. According to equation (20). We identified the model input variables. The results are shown in Table 3.

There are differences in the numerical units and magnitude of different variables. Therefore, the following formula is used to normalize the input variables and output variables of the model to the interval [0, 1], so as to improve the flexibility of data processing:

(21) $$\begin{array}{c} X=\frac{x-x_{\min}}{x_{\max}-x_{\min}}, \end{array}$$

where *x* is the data that needs to be normalized, *X* is the processed data, and *x*_min_ and *x*_max_ are the minimum and maximum values in the dataset, respectively.

### 3.2. GS-ACS-SDBN Prediction Model Construction

Deep neural network can achieve better extraction of feature information, but its multihidden structure leads to its slow learning speed. In this article, the ACS algorithm is used to optimize network weights and deviations to improve the convergence speed and prediction accuracy of SDBN. MAPE is used as the fitness value, and the weight and bias when the training error is the smallest are used as the final parameters of the model.

Before SDBN model training, the model structure parameters need to be set, namely, the number of hidden layers, the number of neurons, and the learning rate. The selection of the above parameters determines the learning ability of the network to the sample features and has an important influence on the prediction accuracy of the model. Therefore, the grid search method is used in this article to determine the optimal combination of the superparameters of the SDBN model. In addition, to avoid the occurrence of overfitting, the 10-fold cross-validation (CV) method was used to suppress the overfitting behavior of the neural network. In the 10-fold cross-validation, the training set was randomly divided into 10 parts, of which 9 parts were used as training samples, and 1 part was used as verification sample. Then, perform 10 times of training, and measure the training error and verification error of the SDBN model with the mean absolute percentage error (MAPE).

The principle of 10-fold cross-validation is shown in Figure 6.

In the process of grid search, different hidden layer numbers and learning rates are combined, and then, 10-fold cross-validation was carried out. Finally, the results of 10-fold cross-validation under different combinations were compared, and the superparameter value corresponding to the minimum error was used as the final selection of the model. The accuracy and the combination of parameters finally selected of grid search for surface roughness, warpage, and tensile strength of FDM parts are shown in Figure 7.

As can be seen from Figure 7, with the increase in the number of hidden layers, the prediction accuracy of the model first increases and then decreases. When the number of hidden layers is less than 4, effective learning of feature information cannot be realized, and the model is in an under-fitting state; when the number of hidden layers is greater than 4, the model has learned too much about data features, and the model is in the fitting state; when the number of hidden layers is set to 4, the prediction accuracy of the model is the highest.

In Figure 7(a), for surface roughness, the optimal combination of hyperparameters *k* = 4 and *ε* = 0.9 is determined, and the training error is 2.07% and the verification error is 3.14%. In Figure 7(b), for the warping degree, the parameter combination is determined as *k* = 4 and *ε* = 0.6 and the training error is 2.15% and the verification error is 3.97%. In Figure 7(c), for the tensile strength, the parameter combination is determined as *k* = 4 and *ε* = 0.7, and the training error is 1.85% and the verification error is 3.53%. At this point, the number of neurons corresponding to each hidden layer is given in Table 4.

Furthermore, we verify the rationality of the above parameter settings based on reconstruction errors, and the results are shown in Figure 8. The results show that the errors of tensile strength, warpage, and roughness can all achieve stability in 100 generations without obvious overfitting behavior.

After the hyperparameters of the SDBN model are determined, we merge the training samples and validation samples; 80% of the training set is reused as the training samples of the SDBN model with the network structure determined, and the ACS algorithm is used to optimize the network learning parameters to obtain the best FDM quality prediction model. The specific process of the SDBN quality prediction model optimized based on ACS algorithm is shown in Figure 9.

## 4. Results and Analysis

In order to test the performance of the model proposed in this article, DBN, RBFNN, LSTM, ANN, and BPNN are used to predict the quality of FDM parts on the same dataset. 10-fold cross-validation and GS are used to determine the hyperparameters of the above models. We retained the model corresponding to the hyperparameter with the highest prediction accuracy and then imported the complete training set to train the model, so as to determine the final prediction model and realize the prediction of the three quality characteristics of FDM parts. The training errors and validation errors of the 10-fold cross-validation of different models are shown in Figure 10.  Table 5 shows the error statistical results of all the prediction models.

Cross-validation can be used not only for parameter adjustment, but also for model evaluation. In Figure 10, we compared the training error and validation error of different models for 10 times of 10-fold cross-validation. The results in the figure show that the 10-fold cross-validation training error results of the GS-ACS-SDBN, DBN, RBFNN, LSTM, and BPNN models can maintain relatively stable results. Among them, the GA-ACS-SDBN model 10-fold cross-validation training results are optimal. On the validation set, compared to the stable results of the GS-ACS-SDBN and DBN models, the 10-fold cross-validation errors of the RBFNN, LSTM, and BPNN models show significant differences. Furthermore, according to the statistical results of 10-fold cross-validation errors in Table 5, the average values of the 10-fold cross-validation training errors of the GS-ACS-SDBN model for the tensile strength, curvature, and surface roughness of FDM parts are 2.02%, 2.10%, and 1.95% respectively. The mean values of 10-fold cross-validation errors were 3.43%, 4.08%, and 3.03%, respectively. Compared with DBN, RBFNN, LSTM, and BPNN, the accuracy of the proposed model is significantly improved, and the stability of the model is strong.

We retained the network parameters with the least error in the 10-fold cross-validation, then input the entire training set into the debugged model for training, and evaluated the model on the test set.  Table 5 compares the training error and test error of tensile strength, warpage, and surface roughness of FDM parts under different models. From the experimental results, in terms of training errors, the training errors of the GS-ACS-SDBN model for the three quality characteristics are 1.82%, 1.95%, and 2.14, respectively. Compared with the DBN model, the GS-ACS-SDBN improved by 0.95%, 0.78%, and 0.67%. Compared with the LSTM model, it increased by 1.00%, 1.36%, and 1.52%. Compared with the RBFNN model, the results were improved by 1.86%, 2.01%, and 2.38%. Compared with the BPNN model, it improved by 1.80%, 2.58%, and 2.63%. The above results show that the GS-ACS-SDBN model can learn the sample features more fully and obtain better training errors. In terms of test error, the GS-ACS-SDBN model still maintains its superior predictive ability. The prediction errors of tensile strength, warpage, and surface roughness of FDM parts under this model are 2.35%, 3.33%, and 2.64%, respectively. It is 1.27%, 1.28%, and 1.88% higher than the DBN model; 2.19%, 2.70%, and 3.03% higher than the LSTM model; 3.70%, 3.84%, and 3.58% higher than the RBFNN model; and 4.09%, 4.14%, and 3.86% higher than the BPNN model. The above results further indicate that the GS-ACS-SDBN model designed in this article has stronger feature learning ability and mapping ability and can achieve accurate prediction between FDM process parameters and part quality characteristics, showing better prediction performance.

In addition, due to the introduction of the adaptive cuckoo search algorithm, the GS-ACS-SDBN model can optimize network parameters in a relatively short period of time, complete model training in 35.37 s, and output prediction results in 2.44 s. Comparison curves of actual and predicted values of 500 groups of test samples under different models are shown in Figure 11. It can be seen from Figure 11 that compared to DBN, LSTM, RBFNN and BPNN, the change trend of the predicted value of the GS-ACS-SDBN model is almost the same as the real value, and the curve overlap is the highest. The experimental results fully demonstrate the effectiveness and superiority of the ACS-SDBN model in predicting the tensile strength, warping degree, and surface roughness of FDM parts.

## 5. Conclusion

There are complex nonlinear relations between the quality of FDM parts and various process parameters, and it is difficult to predict accurately by traditional methods. In order to solve this problem, based on the DBN, this article establishes a mixed quality prediction model (GS-ACS-SDBN) based on deep learning. The digital prediction of tensile strength, warpage, surface roughness, and other quality characteristics of FDM parts under the influence of multiple process parameters is realized. The research conclusions are as follows:

1. The correlation analysis method (RV_mod_) was used to determine the key quality factors affecting surface roughness, including slice thickness, nozzle temperature, extrusion speed, tensile strength, and material density. The section thickness, nozzle temperature, melting temperature, and bending modulus are the key factors affecting the warpage degree; section thickness, nozzle temperature, extrusion speed, and molding room temperature are the key qualities affecting tensile strength.
2. Based on the 10-fold cross-validation and GS method, the optimal hidden layer of the network is determined to be 4, and the optimal validation errors of roughness, warpage, and tensile strength of FDM parts are 3.14%, 3.97%, and 3.53%, respectively. The reconstruction errors of training samples reach a stable state within 100 iterations.
3. The proposed model is applied to the quality prediction of FDM parts. The experimental results show that the prediction accuracy, stability, and convergence speed of the GS-ACS-SDBN model for tensile strength, warping degree, and surface roughness of FDM parts are better than DBN, LTSM, RBFNN, and BP models. The CV verification error of the model in this article is within 4.08%, and the prediction error is within 3.33%.

The research contents of this article can provide effective research ideas for the application of the GS-ACS-SDBN prediction model in other fields. For different application fields, different sample data are used to train and construct the SDBN model. GS and ACS algorithm are used to optimize network parameters and obtain the best prediction model.

## Figures and Tables

**Figure 1:** RBN structure and DBN structure.

**Figure 2:** Levy flight path.

**Figure 3:** The quality prediction process of FDM parts based on the GS-ACS-SDBN model.

**Figure 4:** FDM parts forming process.

**Figure 5:** FDM parts printing pattern.

**Figure 6:** Schematic of 10-fold cross-validation.

**Figure 7:** Hyperparameter grid search results.

**Figure 8:** Relationship between the reconstruction errors of surface roughness, warpage, and tensile strength and the number of iterations.

**Figure 9:** The specific process of the SDBN quality prediction model optimized based on the ACS algorithm.

**Figure 10:** 10-folding cross-validation calculation process.

**Figure 11:** Comparison of predicted and actual values of tensile strength, warpage, and surface roughness of FDM part.

**Algorithm 1:** RBM training.

**Algorithm 2:** ACS Algorithm.

**Table 1:** FDM process parameters.

Process parameters	Numerical range
Slice thickness	0.05–0.2 mm
Extrusion speed	10–50 mm/s
Nozzle temperature	220–270°C
Molding room temperature	24.2–35.5°C

**Table 2:** Material performance parameters.

Materials	ABS	PLA
Melting temperature	220–250°C	190–220°C
Tensile strength	>43 MPa	>60 MPa
Bending modulus	>60 MPa	>60 MPa
Density	1.04 g/cm^3^	1.25 g/cm^3^
Water imbibition	10%	3%

**Table 3:** Correlation degree between key quality factors and each quality characteristic.

Model input variables	Quality index	RV_mod_
Slice thickness, nozzle temperature, extrusion speed, tensile strength, material density	Surface roughness	0.785
Slice thickness, nozzle temperature, melting temperature, bending modulus	Warping degree	0.722
Slice thickness, nozzle temperature, extrusion speed, and molding room temperature	Tensile strength	0.7593

**Table 4:** The number of neurons contained in each hidden layer.

Quality characteristics	Number of neurons in each hidden layer *n*_*k*_			
	*n*_1_	*n*_2_	*n*_3_	*n*_4_
Surface roughness	8	15	7	4
Warping degree	8	17	11	7
Tensile strength	6	13	9	5

**Table 5:** Error results and running time statistics for different models.

Quality characteristics	Prediction model	CV training error (%)	CV validation error (%)	Training error (%)	Test error (%)	Training time/s	Test time/s
Tensile strength/MPa	GS-ACS-SDBN	2.02	3.43	1.82	2.35	35.37	2.44
	DBN	2.85	4.26	2.77	3.61	88.09	5.82
	LSTM	2.80	4.94	2.82	4.54	42.66	4.13
	RBFNN	4.05	6.28	3.68	6.05	48.31	4.85
	BPNN	4.69	7.00	3.62	6.44	57.85	3.92

Warping degree/mm	GS-ACS-SDBN	2.10	4.08	1.95	3.33	35.37	2.44
	DBN	2.87	4.88	2.73	4.61	88.09	5.82
	LSTM	3.13	6.51	3.31	6.04	42.66	4.13
	RBFNN	4.10	7.36	3.96	7.18	48.31	4.85
	BPNN	4.77	7.54	4.53	7.47	57.85	3.92

Surface roughness/um	GS-ACS-SDBN	1.95	3.03	2.14	2.64	35.37	2.44
	DBN	3.03	4.72	2.81	4.51	88.09	5.82
	LSTM	3.65	6.71	3.66	5.67	42.66	4.13
	RBFNN	4.31	7.74	4.52	6.22	48.31	4.85
	BPNN	4.95	7.74	4.77	6.50	57.85	3.92

## Data Availability

The data used in this article cannot be provided for the following reasons: (1) the parameters in this article are derived from product research and development, and the processing process is confidential; (2) next, the process needs to apply for a patent for invention; and (3) the experimental data will play an important role in the further research.
